The article "Macrophage Rmp Ameliorates Myocardial Infarction by Modulating Macrophage Polarization in Mice" was retracted in 2024. Reasons: signs of a paper mill; compromised peer review; unreliable results or conclusions.

# Macrophage Rmp Ameliorates Myocardial Infarction by Modulating Macrophage Polarization in Mice

**DOI:** 10.1155/2022/6248779

**Published:** 2022-09-01

**Authors:** Jian Zhang, Zongtao Yin, Liming Yu, Zhishang Wang, Yu Liu, Xiaoru Huang, Song Wan, Hui-yao Lan, Huishan Wang

**Affiliations:** ^1^Department of Cardiovascular Surgery, General Hospital of Northern Theater Command, No. 83, Wenhua Road, Shenhe District, Shenyang, Liaoning, China; ^2^Department of Medicine & Therapeutics, and Li Ka Shing Institute of Health Sciences, The Chinese University of Hong Kong, Shatin, NT, Hong Kong; ^3^Division of Cardiothoracic Surgery, Department of Surgery, The Chinese University of Hong Kong, Prince of Wales Hospital, Shatin, NT, Hong Kong

## Abstract

**Background:**

Inflammation plays important roles during myocardial infarction (MI). Macrophage polarization is a major factor that drives the inflammatory process. Our previous study found that RNA polymerase II subunit 5-mediating protein (RMP) knockout in cardiomyocytes caused heart failure by impairing mitochondrial structure and function. However, whether macrophage RMP plays a role in MI has not been investigated.

**Methods:**

Macrophage RMP-knockout in combination with a mouse model of MI was used to study the function of macrophage RMP in MI. Next, we modified bone marrow-derived macrophages (BMDMs) by plasmid transfection, and the BMDMs were administered to LysM-Cre/DTR mice by tail vein injection. Immunoblotting and immunofluorescence were used to detect macrophage polarization, fibrosis, angiogenesis, and the p38 signaling pathway in each group.

**Results:**

Macrophage RMP deficiency aggravates cardiac dysfunction, promotes M1 polarization, and inhibits angiogenesis after MI. However, RMP overexpression in macrophages promotes M2 polarization and angiogenesis after MI. Mechanistically, we found that RMP regulates macrophage polarization through the heat shock protein 90– (HSP90–) p38 signaling pathway.

**Conclusions:**

Macrophage RMP plays a significant role in MI, likely by regulating macrophage polarization via the HSP90–p38 signaling pathway.

## 1. Introduction

Myocardial infarction (MI) is a serious ischemic heart disease caused by atherosclerosis and is associated with high morbidity and mortality rates [1]. Following infarction, cardiomyocyte death and acute inflammation are induced [2]. Inflammation plays important roles during MI [3, 4]. Macrophage polarization is considered to be a major factor that drives the inflammatory process [3]. Macrophages are generally divided into two groups: the classically activated (M1) macrophages and the alternatively activated (M2) macrophages [5, 6]. M1 macrophages could degrade the extracellular matrix and get rid of cell debris; in contrast, M2 macrophages promote the production of anti-inflammatory cytokines, angiogenesis, and collagen deposition [7]. Therefore, targeting macrophage-mediated inflammatory reactions may be an attractive approach to ameliorate MI.

The article "Macrophage Rmp Ameliorates Myocardial Infarction by Modulating Macrophage Polarization in Mice" was retracted in 2024. Reasons: signs of a paper mill; compromised peer review; unreliable results or conclusions.

RNA polymerase II subunit 5-mediating protein (RMP), also known as unconventional prefoldin RPB5 interactor, is widely studied in several types of malignant tumors [8–13]. Some studies showed that RMP could interact with heat shock protein 90 (HSP90) and the R2TP/prefoldin-like complex, which assembles RNA polymerase II before its nuclear translocation [14]. We previously showed that RMP levels are significantly decreased in the cardiomyocytes of patients with heart failure compared with their levels in normal cardiac tissues [15]. Mechanistically, RMP-knockout in cardiomyocytes causes heart failure by impairing mitochondrial structure and function [15]. However, whether macrophage RMP plays a role in MI and how RMP affects macrophage phenotypes have not been investigated.

## 2. Materials and Methods

This research fully complied with ethics guidelines. All animal experiments were performed following the NIH guidelines (*Guide for the Care and Use of Laboratory Animals*) and the ARRIVE guidelines. All experiments were conducted in accordance with the protocols approved by the Institutional Animal Care and Use Committee of the General Hospital of the Northern Theater Command (No. 2015023).

### 2.1. Human Heart Tissue

Ischemic failure hearts from patients who underwent heart transplantation were collected from the General Hospital of the Northern Theater Command, Shenyang, China. This study was approved by the Ethics Committee of the General Hospital of the Northern Theater Command (No. 2015103). All participants provided written informed consent.

### 2.2. MI Mouse Model

MI was induced by ligation of the left main descending coronary artery as described previously [16]. Briefly, mice were anesthetized with ketamine (50 mg/kg) and xylazine (50 mg/kg). The operation was performed under artificial ventilation with respirator support. The left descending coronary artery was ligated using a 6-0 silk suture. Mice in the sham group underwent the same procedure without the ligation step.

### 2.3. Animals

#### 2.3.1. Control and Macrophage-Specific *Rmp*-Knockout Mice

*RMP* ^flox/flox^ mice were generated as described previously [15]. Macrophage-specific *Rmp*-knockout (MRKO) and littermate control (LC) mice were generated by mating *RMP*^flox/flox^ mice with transgenic mice expressing Cre recombinase under the control of the lysozyme M (LysM) promoter. The MRKO and LC mice had a C57BL6 background. Two-month-old age- and weight-matched male LC and MRKO mice were used for the experiments.

The article "Macrophage Rmp Ameliorates Myocardial Infarction by Modulating Macrophage Polarization in Mice" was retracted in 2024. Reasons: signs of a paper mill; compromised peer review; unreliable results or conclusions.

In the macrophage depletion study, macrophages were conditionally deleted from LysM-Cre/diphtheria toxin receptor (DTR) mice by intraperitoneal injection of diphtheria toxin as described previously [16].

### 2.4. Bone Marrow-Derived Macrophage Transplantation

Bone marrow cells were isolated from mice with a C57BL/6J background as described previously [16]. Briefly, bone marrow cells were obtained by flushing the femur and tibia with Dulbecco's modified Eagle's medium/F12 medium. Cell suspensions were collected the next day and further differentiated into macrophages by 5 days of stimulation in Dulbecco's modified Eagle's medium/F12 containing 10% fetal bovine serum and 10 ng/mL macrophage colony-stimulating factor. The bone marrow-derived macrophages (BMDMs) were then transfected with plasmids expressing a short hairpin RNA targeting *Rmp* (shRmp) or *Rmp* according to the manufacturer's protocol. Plasmids expressing shRmp were purchased from GeneChem Co., Ltd. (Shanghai, China), and the plasmid-expressing mouse *Rmp* was kindly provided by Dr. Liwei Dong (International Cooperation Laboratory on Signal Transduction, Eastern Hepatobiliary Surgery Institute, the Second Military Medical University, Shanghai, China). After 24 h of transfection, cell suspensions (1 × 10^6^ cells) were prepared and administered to the LysM-Cre/DTR mice by tail vein injection, 5 days after intraperitoneal injection of diphtheria toxin. Diphtheria toxin was given until cardiac tissues were harvested.

### 2.5. Echocardiography

Transthoracic echocardiography was performed using a Vevo770 high-resolution ultrasound imaging system (VisualSonics, Toronto, Canada) with an RMV 707B scan head (30 MHz, VisualSonics) 1 week after surgery. Mice were anesthetized with ketamine (50 mg/kg) and xylazine (50 mg/kg) on a warming plate to maintain body temperature. Left ventricular internal diameters at end-diastole and end-systole were obtained using M-mode recording. The left ventricular ejection fraction (LVEF) and left ventricular end-diastolic volume (LVEDV) were calculated according to the guidelines of the Vevo770 system (VisualSonics).

### 2.6. Histology

Cardiac tissue sections were prepared and fixed in 4% paraformaldehyde to obtain paraffin-embedded coronal sections for Masson's trichrome staining and immunohistochemical analysis [15]. Masson's trichrome staining (BA4079A; Baso Diagnostics, Zhuhai, China) was performed following the manufacturer's instructions. Immunohistochemical staining was performed using antibodies against RMP (11277-1-AP, 1 : 50; Proteintech, Wuhan, China) and collagen I (1310-01, 1 : 100; Southern Tech, Ardmore, OK, USA). The scar area, intimal area, and medial area were measured using Image-Pro Plus software (Media Cybernetics, Bethesda, MD, USA) [17].

The article "Macrophage Rmp Ameliorates Myocardial Infarction by Modulating Macrophage Polarization in Mice" was retracted in 2024. Reasons: signs of a paper mill; compromised peer review; unreliable results or conclusions.

### 2.7. Immunofluorescence

Periodate–lysine–paraformaldehyde-fixed cardiac tissue was used to prepare frozen sections. RMP was labeled with an anti-RMP antibody (11277-1-AP, 1 : 50, Proteintech). Macrophages in human cardiac tissues were labeled with an anti-CD68 antibody (NB100-683; Novus, Centennial, CO, USA). Nuclei were counterstained with 4′,6-diamidino-2-phenylindole.

### 2.8. Quantitative Reverse Transcription PCR

Total RNA isolation and real-time PCR were performed as described previously [14, 15]. The *Rmp* primer sequences were as follows: forward, 5′-TGCCAAGAGAAAATCCAGCAT-3′; reverse, 5′-AGGTCCTCAGCCTCTCTTGAA-3′.

### 2.9. Western Blot Analysis

Western blot analysis was performed as described previously [15]. Nitrocellulose membranes were incubated overnight at 4°C with diluted antibodies against inducible nitric oxide synthase (iNOS; ab178945; Abcam, Cambridge, UK), cluster of differentiation (CD) 206 (sc-58986; Santa Cruz Biotechnology, Dallas, TX, USA), RMP (11277-1-AP, 1 : 1,000, Proteintech), CD31 (92841; Cell Signaling Technology, Danvers, MA, USA), HSP90AB1 (5087, Cell Signaling Technology), phosphorylated p38 (4511 s, Cell Signaling Technology), or total p38 (8690 s, Cell Signaling Technology). BMDMs were treated with 200 nM 17-allylamino-17-demethoxygeldanamycin (17-AAG; S1141; Selleck, Houston, TX, United States).

### 2.10. Statistical Analysis

The data are presented as mean ± standard error of the mean. Data between groups were compared with an unpaired two-tailed Student's *t* test using Prism 5 (GraphPad Software, La Jolla, CA, USA). Values of *P* < 0.05 were considered statistically significant. Cumulative mortality was analyzed using Kaplan-Meier curves, and a log-rank test was used to assess statistical significance (*P* < 0.05).

## 3. Results

### 3.1. RMP Expression Is Upregulated in Human Macrophages after MI

We first evaluated RMP levels in heart tissue samples from patients with advanced ischemic heart failure who underwent heart transplantation (Table S1). In contrast to the RMP expression level in cardiomyocytes, immunofluorescence showed a significant increase in macrophages of the infarct zone compared with remote areas (Figures 1(a) and 1(b)).

### 3.2. Macrophage RMP Deficiency Aggravates Cardiac Dysfunction after MI

To study the role of macrophage RMP in MI, we generated MRKO mice using the Cre–lox system. BMDMs isolated from LC and MRKO mice were analyzed to assess knockdown efficiency. Owing to the lack of a commercial antibody against mouse RMP [15], *Rmp* mRNA levels were used to validate the knockout model (Figure S1A).

The article "Macrophage Rmp Ameliorates Myocardial Infarction by Modulating Macrophage Polarization in Mice" was retracted in 2024. Reasons: signs of a paper mill; compromised peer review; unreliable results or conclusions.

Next, we induced MI by ligating the left anterior descending artery in LC and MRKO mice. MRKO mice showed a significantly higher mortality rate than LC mice (Figure 2(a)). The hearts of MRKO mice were more dilated than those of LC mice 7 days after MI (Figure 2(b)). Furthermore, the scars were markedly larger in MRKO mice than in LC mice (Figures 2(c) and 2(d)). Echocardiography demonstrated a significant decrease in the LVEF and a significant increase in the LVEDV of MRKO mouse hearts compared with LC mouse hearts (Figures 2(e) and 2(f)). Immunohistochemical analysis also showed that the loss of RMP in macrophages resulted in more severe cardiac fibrosis, as indicated by increased collagen I accumulation at the infarct site in MRKO mice (Figures 2(g) and 2(h)).

### 3.3. Macrophage RMP Deficiency Promotes M1 Polarization and Inhibits Angiogenesis after MI

Studies have shown that macrophage polarization affects infarct healing after MI [3]. Flow cytometry was performed to assess macrophage polarization. The results showed that the expression levels of iNOS (an M1 macrophage marker) were upregulated, while those of CD206 (an M2 macrophage marker) were downregulated in MRKO mice compared with LC mice (Figures 3(a) and 3(b)), suggesting that the deletion of RMP in macrophages promoted M1 macrophage polarization. Western blot analysis confirmed the increase in iNOS expression levels and the decrease in CD206 expression levels in MRKO mice (Figures 3(c) and 3(d)). Angiogenesis is crucial for maintaining cardiac function following MI. We found that the deletion of RMP in macrophages decreased the number of CD31-expressing cells at the infarct site (Figures 3(e) and 3(f)). Moreover, macrophage-specific deletion of RMP downregulated total cardiac expression of CD31 (Figures 3(g) and 3(h)).

### 3.4. RMP in Macrophages Protects against MI

To further assess the role of RMP in macrophages, we used LysM-Cre/DTR mice to delete macrophages. Furthermore, we modified the macrophages by overexpressing or knocking down RMP. The modified macrophages were then administered to LysM-Cre/DTR mice (Figure 4(a)), and the expression of RMP in modified macrophages was detected (Figure S1B). To test this model, we administered BMDMs from Cre-dependent tdTomato reporter transgenic mice [17] to LysM-Cre/DTR mice. Immunofluorescence analysis indicated that most macrophages present were those that were administered (Figure S1C). Mice receiving BMDMs overexpressing RMP (ovRmp BMDMs) showed a clear trend of reduced infarct size compared with mice receiving negative control BMDMs (NC BMDMs) (Figures 4(b) and 4(c)). In contrast, mice receiving RMP knockdown BMDMs (shRmp BMDMs) showed an increased infarct size (Figures 4(b) and 4(c)). RMP overexpression in macrophages improved the LVEF and attenuated dilation (LVEDV, Figures 4(d) and 4(e)). Furthermore, mice with macrophage-specific overexpression of RMP developed mild cardiac fibrosis, as evidenced by a decrease in collagen I accumulation compared with mice receiving NC BMDMs (Figures 4(f) and 4(g)).

The article "Macrophage Rmp Ameliorates Myocardial Infarction by Modulating Macrophage Polarization in Mice" was retracted in 2024. Reasons: signs of a paper mill; compromised peer review; unreliable results or conclusions.

### 3.5. Macrophage RMP Promotes Macrophage M2 Polarization and Angiogenesis after MI

Treatment with ovRmp BMDMs suppressed MI-induced iNOS expression but promoted CD206 expression (Figures 5(a) and 5(b)). Moreover, mice receiving ovRmp BMDMs showed more CD31-positive cells at the infarct site compared with mice receiving NC BMDMs (Figures 5(c) and 5(d)). Furthermore, western blotting analysis also showed that macrophage-specific overexpression of RMP promoted angiogenesis (Figures 5(e) and 5(f)).

### 3.6. RMP Regulates Macrophage Polarization through HSP90-Dependent Mechanisms

Previously, we used label-free mass spectrometry to identify the possible binding proteins of RMP in the AC16 cell line (Table S2). We found that HSP90AB1 is a protein that binds to RMP. This was confirmed by immunofluorescence and co-immunoprecipitation analyses (Figure S1D and E). Several groups have reported that HSP90AB1, along with HSP90AA, modulates macrophage polarization through the p38 mitogen-activated protein kinase (MAPK) pathway [16, 18, 19]. In our mouse model, we also showed that phosphorylated p38 levels were decreased in mice receiving ovRmp BMDMs compared with mice receiving NC BMDMs (Figures 6(a) and 6(b)). In MRKO mice, phosphorylated p38 was upregulated 7 days after MI (Figures 6(c) and 6(d)). Next, we used 17-AAG, a potent HSP90 ATPase inhibitor, to block the effects of HSP90. *In vitro*, RMP overexpression was induced by tumor necrosis factor alpha (TNF-*α*) in BMDMs. We also found that RMP inhibited TNF-*α*-induced iNOS expression and p38 activation, and these effects were blocked by 17-AAG (Figures 6(e)–6(g)).

## 4. Discussion

In this study, we demonstrated that the deletion of RMP in macrophages significantly aggravated myocardial healing after MI in mice. Our findings showed that mice lacking RMP developed more severe MI and showed impaired angiogenesis. Importantly, we also found that RMP overexpression in macrophages improved post-MI cardiac physiology and increased cardiac M2 macrophage polarization.

Our data identified macrophage RMP as a promising new target for treating MI. Following MI, the death of cardiomyocytes causes an immune response that leads to further tissue destruction [5]. Macrophages have been recognized as important regulators of and participants in inflammation and fibrosis following MI. In the initial stage of MI, the injured heart is dominated by proinflammatory (M1) macrophages, whereas several days later, macrophages with an anti-inflammatory phenotype (M2) become predominant. Several studies have indicated that M2-like macrophages are beneficial for cardiac tissue repair [20]. Therefore, therapeutic strategies that promote M2 polarization of MI macrophages may also promote myocardial repair. Macrophage RMP deficiency has been shown to aggravate MI, especially because the effects of RMP are cardioprotective, by shifting proinflammatory cardiac M1 macrophages to the reparative M2 phenotype. Indeed, macrophage RMP exerts its inhibitory effect on macrophage activation via the p38 MAPK signaling pathway. Understanding this mechanism may help us develop novel treatment strategies for ischemic heart disease. However, effective and safe ways to deliver inhibitors or purified protein to the infarction area are still lacking. Percutaneous coronary intervention may be the optimal way to deliver drugs, inhibitors, or purified protein for treating MI.

The article "Macrophage Rmp Ameliorates Myocardial Infarction by Modulating Macrophage Polarization in Mice" was retracted in 2024. Reasons: signs of a paper mill; compromised peer review; unreliable results or conclusions.

As an oncogene, *Rmp* is amplified and overexpressed in many malignancies, such as ovarian cancer [21], hepatocellular carcinoma [9, 12], prostate cancer [22], cholangiocarcinoma [13], and colorectal cancer [23]. Our previous study found that cardiomyocyte-specific knockout of *Rmp* results in contractile dysfunction, cardiac dilatation, and fibrosis owing to impaired mitochondrial structure and function through the regulation of peroxisome proliferator-activated receptor-gamma coactivator alpha-dependent mitochondrial function via a transforming growth factor-beta/mothers against the decapentaplegic homolog 3-dependent mechanism [15]. RMP is a transcription-mediating protein that binds with RNA polymerase II subunit 5 [9]. Mass spectrometry results showed that HSP90AB1 is a potential RMP-binding protein. Moreover, co-immunoprecipitation analysis confirmed the binding between RMP and HSP90AB1. In line with our findings, RMP, as part of a protein complex known as the R2TP/prefoldin-like complex, along with HSP90, has been shown to be responsible for the cytoplasmic assembly of RNA polymerase II [14, 24]. HSP90 proteins constitute a family of highly conserved molecular chaperones that modulate the biological activities of their client proteins. It has been reported that HSP90 participates in macrophage activation [25]. In intervertebral disc degeneration, the HSP90 inhibitor 17-AAG attenuates the proinflammatory activity of M1 macrophages by inhibiting the p38 MAPK pathway. HSP90 has been reported to be essential for iNOS (M1 marker) gene transactivation [26]. Here, we found that RMP overexpression inhibited iNOS expression in BMDMs, but HSP90 inhibition with 17-AAG upregulated the iNOS expression inhibited by RMP. We found that the p38 MAPK pathway was the possible signaling pathway modulating the effects of RMP on macrophage polarization.

The article "Macrophage Rmp Ameliorates Myocardial Infarction by Modulating Macrophage Polarization in Mice" was retracted in 2024. Reasons: signs of a paper mill; compromised peer review; unreliable results or conclusions.

As an oncogene, *Rmp* has been reported to promote venous invasion and vascularization [9, 10]. However, angiogenesis benefits cardiac tissue repair after MI. Our data showed that RMP in macrophages promotes angiogenesis after MI. This finding is consistent with the proangiogenic effect of RMP in many malignancies. Furthermore, RMP, along with HSP90AB1 and HSP90AA, may be involved in regulating protein expression. Hypoxia-inducible factor- (HIF-) 1*α* is a master transcriptional factor for angiogenesis during cardiac repair, and Hsp90 has been reported to stabilize HIF-1*α* [27, 28]. The binding between RMP and HSP90 observed in our study may also indicate that RMP participates in the regulation of HIF-1*α* expression after MI. However, the underlying mechanism whereby macrophage RMP promotes angiogenesis was not fully elucidated.

## 5. Conclusion

In summary, macrophage RMP plays a significant role in MI, likely by regulating macrophage polarization via the HSP90–p38 signaling pathway. These results have uncovered a novel function of macrophage RMP in MI, and they support the selective targeting of RMP in macrophages as an effective novel strategy to treat MI.

## Figures and Tables

**Figure 1:** RMP expression is upregulated in human macrophages after myocardial infarction. (a) Representative immunofluorescence staining of RNA polymerase II subunit 5-mediating protein (RMP, red) and CD68 (green) from patients with advanced ischemic heart failure. Scale bar = 100 *μ*m. (b) Quantification of both RMP- and CD68-positive cells.

**Figure 2:** Macrophage Rmp deficiency aggravates cardiac dysfunction after myocardial infarction. (a) Survival curves for macrophage-specific Rmp-knockout (MRKO) and littermate control (LC) mice. ^∗∗∗^*P* < 0.001. *N* = 15 mice per group. (b) Representative images of the hearts from LC and MRKO mice collected 7 days after myocardial infarction (MI). Scale bar = 2 mm. (c) Representative images of infarct size after Masson's trichrome staining of the hearts collected 7 days after the induction of MI. (d) Quantification of fibrosis as a percentage of total myocardial tissue area. Values are mean ± SEM of *n* = 6 per group. Student's *t* test, ^∗^*P* < 0.05. (e) Representative echocardiography (M-mode) and left ventricular function 7 days after the induction of MI. (f) Echocardiographic analysis of LVEF and LVEDV (*n* = 5; Student's *t* test, ^∗∗∗^*P* < 0.001). (g) Immunohistochemical staining of collagen I accumulation at the infarct site 7 days after the induction of MI. Scale bar = 200 *μ*m. (h) Quantitative analysis of collagen I (*n* = 5; Student's *t* test, ^∗∗∗^*P* < 0.001).

The article "Macrophage Rmp Ameliorates Myocardial Infarction by Modulating Macrophage Polarization in Mice" was retracted in 2024. Reasons: signs of a paper mill; compromised peer review; unreliable results or conclusions.

**Figure 3:** Macrophage Rmp deficiency promotes M1 polarization and inhibits angiogenesis after myocardial infarction. (a) Three-color flow cytometry shows the M1 (CD68+/iNOS+) and M2 (CD68+/CD206+) macrophages at the infarct site 7 days after myocardial infarction (MI). (b) Quantitative analysis of M1 and M2 macrophages (*n* = 5; Student's *t* test, ^∗∗∗^*P* < 0.001). (c) Representative images of CD206 and iNOS by western blotting 7 days after MI. (d) Corresponding densitometric quantification of the immunoreactive bands. Values are mean ± SEM of *n* = 5 per group. ^∗∗∗^*P* < 0.001 versus LC by unpaired Student's. (e) Two-color immunofluorescence shows CD31 in LC and MRKO mice 7 days after MI. (f) Quantitative analysis of CD31. Values are mean ± SEM of *n* = 5 per group. ^∗∗∗^*P* < 0.001 versus LC by unpaired Student's. (g) Representative images of CD31 in the infarct area of LC and MRKO mice by western blotting 7 days after MI. (h) Quantitative analysis of CD31. Values are mean ± SEM of *n* = 5 per group. ^∗∗∗^*P* < 0.001 versus LC by unpaired Student's.

**Figure 4:** Macrophage Rmp protects against myocardial infarction. (a) Study design of bone marrow transplantation experiments, in which the mice were induced MI. (b) Representative images of infarct size by Masson's trichrome staining 7 days after MI. (c) Quantitative analysis of fibrosis as a percentage of total myocardial tissue area. *n* = 4–6 per group. Values are mean ± SEM. Student's *t* test, ^∗∗^*P* < 0.01. (d) Representative echocardiography (M-mode) 7 days after MI. (e) Echocardiographic analysis of LVEF and LVEDV (*n* = 5; Student's *t* test, ^∗^*P* < 0.05 and ^∗∗^*P* < 0.01). (f) Immunohistochemical staining of collagen I accumulation at the infarct site 7 days after MI. Scale bar = 200 *μ*m. (g) Quantitative analysis of collagen I (*n* = 5; Student's *t* test, ^∗^*P* < 0.05).

**Figure 5:** Macrophage Rmp promotes macrophage M2 polarization and angiogenesis after myocardial infarction. (a) Representative images of CD206 and iNOS by western blotting 7 days after myocardial infarction (MI). (b) Corresponding densitometric quantification of the immunoreactive bands. Values are mean ± SEM of *n* = 4 − 6 per group. ^∗^*P* < 0.05, ^∗∗^*P* < 0.01, and ^∗∗∗^*P* < 0.001 by unpaired Student's. (c) Two-color immunofluorescence analysis shows CD31 in mice receiving the indicated bone marrow-derived macrophages (BMDMs) 7 days after MI. (d) Quantitative analysis of CD31. Values are mean ± SEM of *n* = 5 per group. ^∗^*P* < 0.05, ^∗∗^*P* < 0.01, and ^∗∗∗^*P* < 0.001 by unpaired Student's. (e) Representative image analysis of CD31 in the infarct area of mice receiving the indicated BMDMs by western blotting 7 days after MI. (f) Quantitative analysis of CD31. Values are mean ± SEM of *n* = 5 per group. ^∗^*P* < 0.05, ^∗∗^*P* < 0.01, and ^∗∗∗^*P* < 0.001 by unpaired Student's.

The article "Macrophage Rmp Ameliorates Myocardial Infarction by Modulating Macrophage Polarization in Mice" was retracted in 2024. Reasons: signs of a paper mill; compromised peer review; unreliable results or conclusions.

**Figure 6:** Rmp regulates macrophage polarization through heat shock protein 90-dependent mechanisms. (a) Representative image and quantitative analysis of phosphorylated (p-) p38 and nonphosphorylated p38 in the infarct area of mice by western blotting 7 days after myocardial infarction (MI). (b) Corresponding densitometric quantification of the immunoreactive bands. Values are mean ± SEM of *n* = 4 − 6 per group. ^∗^*P* < 0.05 and ^∗∗^*P* < 0.01, by unpaired Student's. (c) Representative image analysis of p-p38 and p38 in the infarct area of littermate control (LC) and macrophage-specific Rmp-knockout (MRKO) mice by western blotting 7 days after MI. (d) Quantitative analysis of p-p38. Values are mean ± SEM of *n* = 5 per group. ^∗^*P* < 0.05, by unpaired Student's. (e) Representative images analysis of p-p38 and p38 in bone marrow-derived macrophages by western blotting. (f and g) Quantitative analysis of iNOS and p-p38. Values are mean ± SEM of *n* = 5 per group. ^∗^*P* < 0.05; ns, *P* > 0.05 by unpaired Student's.

## Data Availability

The data used to support the findings of this study are available from the corresponding author upon request.

## Abbreviations

MI: Myocardial infarction
RMP: RNA polymerase II subunit 5-mediating protein
BMDM: Bone marrow-derived macrophage
Hsp90: Heat shock protein 90
MRKO: Macrophage-specific *Rmp-*knockout
LC: Littermate control
LysM: Lysozyme M
DTR: Diphtheria toxin receptor
LVEF: Left ventricular ejection fraction
LVEDV: Left ventricular end-diastolic volume
MAPK: Mitogen-activated protein kinase
TNF-*α*: Tumor necrosis factor alpha.

## Supplementary Materials

Supplementary 1 Figure S1: (A) relative expression of Rmp in BMDM from LC and MRKO mice. (B) Relative expression of Rmp in modified BMDM. (C) Representative immunofluorescence staining of F4/80 (green) and Tomato from DTR mice receiving BMDM of Cre-dependent tdTomato. (D) Representative immunofluorescence staining of RMP (green) and HSP90AB1 (red) in AC16 cell. (E) AC16 cells were harvested. Whole-cell lysates were immunoprecipitated with RMP or HSP90AB1 antibody respective or control immunoglobulin G and analyzed by western blotting. Cell lysates were also subjected to immunoblotting. (F) Relative expression of TNF-*α* and IL-6 in BMDM from LC and MRKO mice under the treatment of LPS (upper). Relative expression of TNF-*α* and IL-6 in overexpressed Rmp BMDM (lower).

The article "Macrophage Rmp Ameliorates Myocardial Infarction by Modulating Macrophage Polarization in Mice" was retracted in 2024. Reasons: signs of a paper mill; compromised peer review; unreliable results or conclusions.

Supplementary 2 Table S1: clinical characteristics pertaining to patients with ischemic heart failure.

Supplementary 3 Table S2: label-free mass spectrometry identified the possible binding proteins of RMP in the AC16 cell line.
